# Continuity of Care plus Whole Process Psychological Intervention for Lung Cancer Patients undergoing Chemotherapy

This article has been retracted.

**DOI:** 10.1155/2022/4330059

**Published:** 2022-04-21

**Authors:** Chunxiang Zhou, Jinghua Tang, Fenlan Sun, Lei Huang, Mengyue Liu, Dan Kuang

**Affiliations:** ^1^Department of Respiratory Medicine, Affiliated Hospital of Jiangnan University, Wuxi, China; ^2^Department of Nursing, Affiliated Hospital of Jiangnan University, Wuxi, China

## Abstract

**Objective:**

To explore the efficiency of continuity of care plus whole process psychological intervention for lung cancer patients undergoing chemotherapy.

**Methods:**

A total of 130 patients who have lung cancer undergoing chemotherapy admitted to our hospital from 2019 to 2021 were recruited and assigned via different intervention methods (1 : 1) to receive either continuity of care plus whole process psychological intervention (observation group) or routine nursing (control group). Outcome measures included psychological state, treatment compliance, quality of life, and nursing satisfaction.

**Results:**

Continuity of care plus whole process psychological intervention was associated with significantly lower Hamilton Depression Scale (HAMD) and Hamilton Anxiety Scale (HAMA) scores versus routine care. The patients given combined nursing showed higher self-esteem scores versus those given routine care. Continuity of care plus whole process psychological intervention also resulted in significantly lower cancer-related fatigue scores and higher treatment compliance versus routine care. Patients given continuity of care plus whole process psychological intervention had a better quality of life and higher nursing satisfaction versus those given routine care (*P* < 0.05).

**Conclusions:**

Continuity of care plus whole process psychological intervention can effectively mitigate the negative emotions of lung cancer patients, alleviate cancer-related fatigue, improve treatment compliance, and boost the life quality of patients.

## 1. Introduction

Lung cancer ranks top in the incidence and mortality of malignancies in China [1]. Current clinical treatment methods include surgery, radiotherapy, and chemotherapy. Chemotherapy can inhibit the growth of cancer cells but may result in collateral damage to adjacent normal cells, which elicits multiple complications after treatment [2]. It has been reported that lung cancer patients after chemotherapy are prone to adverse psychological states such as depression, anxiety, fatigue, and irritability [3, 4]. Moreover, lax treatment compliance may cause disease recurrence [5]. Routine care only covers patients' stay in hospitals [6, 7], while the whole process psychological intervention allows postdischarge care of patients, which provides an extended professional nursing session for a better recovery of patients [8]. Continuity of care is an extension of inpatient nursing based on holistic nursing theory and humanistic care theory and ensures the nursing quality after discharge to promote rehabilitation and avoid readmission [9], thereby enhancing the quality of life of patients [10, 11]. Accordingly, the present study was conducted to explore the efficiency of continuity of care plus whole process psychological intervention for lung cancer patients undergoing chemotherapy.

## 2. Materials and Methods

### 2.1. General Data

In this retrospective study, 130 lung cancer patients undergoing chemotherapy admitted to our hospital from 2019 to 2021 were randomly enrolled and assigned to the observation group (*n* = 65) and control group (*n* = 65) based on different nursing care methods. The protocol was approved by the Affiliated Hospital of Jiangnan University (no. JN3297-091). All subjects gave written informed consent in accordance with the Declaration of Helsinki.

### 2.2. Inclusion and Exclusion Criteria

Inclusion criteria are as follows: (1) all patients were diagnosed with lung cancer by pathology; (2) with the first onset; and (3) the patients were informed of the study and provided written informed consent.

Exclusion criteria are as follows: (1) patients with disturbance of consciousness or serious diseases of important organs; (2) with an estimated survival of less than half a year; and (3) with coagulation dysfunction.

### 2.3. Nursing Methods

The control group patients received routine nursing, including medication instruction, health education, diet instruction, and life behavior guidance. The patients were given nursing instructions and precautions for self-care after discharge. Telephone follow-up was performed once a week after discharge.

The patients in the observation group received continuity of care plus whole process psychological intervention: (1) a continuity of care group was established and all nurses were systematically trained. (2) A targeted nursing plan was formulated according to the actual situation of the patient. (3) Medical support was provided timely to address adverse reactions during home care, and active communication with the patients was conducted to supervise the patients' psychological status. (4) The disease conditions were followed up regularly with feedback from the patients. The patients were also given diet and exercise guidance and were encouraged to participate in social activities to maintain a positive treatment attitude [12]. (5) Health education was performed to enhance the patients' awareness of the disease and reduce negative emotions. (6) Analgesic drugs were given to patients with severe pain.

### 2.4. Evaluation Criteria

1. Hamilton Depression Scale (HAMD) and Hamilton Anxiety Scale (HAMA) were used to evaluate the depression and anxiety of the two groups before and after the intervention. HAMD includes 24 items and HAMA includes 14 items. The score is proportional to the depression and anxiety of the patients.
2. The self-esteem scale (SES) evaluates the self-esteem of patients. The scale is composed of 5 positive scores and 5 reverse scores. A score less than 15 indicates an inferiority complex.
3. The cancer-related fatigue was evaluated in four dimensions of body, cognition, behavior, and emotion after discharge, with a score ranging from 0 to 10 points for each dimension. The higher the score, the more severe the fatigue.
4. Morisky Compliance Scale was used to evaluate the treatment compliance of patients before and after nursing intervention from the following four aspects: medication compliance, body weight control, diet control, and appropriate exercise, with a full score of 50 points. 50 points: good compliance; 30–40: partial compliance; <30 points: poor compliance.
5. The life quality of patients after discharge was assessed by the lung cancer life quality assessment scale (Chinese version), which was divided into five dimensions, including lung cancer-specific module, functional dimension, physiological dimension, social/family dimension, and emotional dimension. The score of each dimension is 0–10 points, and the score is proportional to the life quality.
6. The nursing satisfaction questionnaire created by our hospital is divided into highly satisfied, satisfied, less satisfied, and dissatisfied.

### 2.5. Data Analysis

GraphPad Prism 8 software is used to process images, and SPSS22.0 software is used for data analyses. Count data are expressed as (*n* (%)) and analyzed by the chi-square test, and measurement data are expressed as ($\bar{x}\pm s$) and processed by the *t*-test. Differences are considered statistically significant at *P* < 0.05.

## 3. Results

### 3.1. General Data

The observation group included 39 males and 26 females, aged 41–78 (58.89 ± 12.13) years. There were 11 cases of small cell lung cancer, 21 cases of squamous cell carcinoma, 27 cases of adenocarcinoma, 6 cases of large cell carcinoma, 35 cases of TNM stage III, and 30 cases of TNM stage IV. The control group had 41 males and 24 females, aged 42–79 (58.76 ± 12.57) years, including 9 cases of small cell lung cancer, 19 cases of squamous cell carcinoma, 32 cases of adenocarcinoma, 5 cases of large cell carcinoma, 32 cases of TNM stage III and 33 cases of TNM stage IV. There was no significant difference in the general data between these two groups (*P* > 0.05, Table 1).

### 3.2. Depression and Anxiety

Before nursing, there was no significant difference in HAMD and HAMA scores between the two groups (*P* > 0.05). The HAMD and HAMA scores of the two groups after nursing intervention were lower than those before the nursing. The HAMD and HAMA scores of the patients in the observation group (18.25 ± 3.45, 12.66 ± 2.14) were significantly lower than the patients in the control group (25.68 ± 4.69, 16.73 ± 3.64) (*P* < 0.05, Table 2).

### 3.3. Self-Esteem Scores

There was no significant difference in self-esteem psychology between the two groups before nursing (*P* > 0.05). After nursing, the psychological scores of self-esteem were improved, and the psychological scores of self-esteem in the observation group (25.69 ± 4.36) were higher than those in the control group (19.12 ± 3.65) (*P* < 0.05, Figure 1).

### 3.4. Cancer-Related Fatigue

After nursing, the scores of physical dimension, behavioral dimension, cognitive dimension, and emotional dimension (5.39 ± 0.13, 3.08 ± 0.52, 3.43 ± 0.49 and 4.28 ± 0.74) in the observation group were lower than those in the control group (7.13 ± 1.28, 4.83 ± 1.17, 4.71 ± 1.23, and 6.23 ± 0.68) (*P* < 0.05, Table 3).

### 3.5. Treatment Compliance

There was no significant difference in the Morisky score between the two groups before nursing (*P* > 0.05). After nursing, the Morisky scores of the two groups were improved, and the observation group showed higher results (28.34 ± 3.49, 30.01 ± 3.65, 31.65 ± 4.23, and 31.56 ± 4.18) than the control group (38.32 ± 2.13, 42.91 ± 2.98, 41.28 ± 1.79, and 40.08 ± 3.89) (*P* < 0.05, Figure 2).

### 3.6. Life Quality Score

After the nursing, the scores of lung cancer-specific module, functional dimension, social/family dimension, emotional dimension, and physiological dimension (25.18 ± 1.62, 23.58 ± 3.15, 25.54 ± 2.37, 21.35 ± 0.49, and 25.32 ± 3.23) in the observation group were higher than those in the control group (33.70 ± 1.31, 17.24 ± 1.33, 20.08 ± 1.64, 17.36 ± 0.14, and 18.04 ± 0.39) (*P* < 0.05, Table 4).

### 3.7. Nursing Satisfaction

The observation group had 38 (58.46%) cases of highly satisfied, 26 (40.00%) cases of satisfied, 1 (1.54%) case of less satisfied, and 0 (0.00%) of dissatisfied, with the total satisfaction of 98.46%. The control group had 18 (27.69%) cases of highly satisfied, 24 (36.93%) cases of satisfied, 17 (26.15%) cases of less satisfied, and 6 (9.23%) cases of dissatisfied, with the total satisfaction of 64.62%. A significantly higher satisfaction was observed in the observation group versus the control group (*P* < 0.05, Figure 3).

## 4. Discussion

Lung cancer is a malignancy with the highest incidence and mortality worldwide [13,14]. Current clinical treatment methods include surgery, radiotherapy, and chemotherapy. Despite a promising efficacy in cancer cell growth inhibition, chemotherapy may cause collateral damage to normal cells and lead to adverse events [15]. Continuity of care refers to targeted nursing schemes to ensure professional and effective nursing care at hospitals and homes. The whole process psychological intervention allows extended nursing care after discharge to enhance the nursing efficiency [16, 17]. The results by Jahn et al. showed that after the psychological intervention, the cancer recurrence and mortality of cancer patients were decreased, which was consistent with the results of the present study [18, 19].

Here, continuity of care plus whole process psychological intervention was associated with significantly lower HAMD and HAMA scores and higher self-esteem scores versus routine care. Continuity of care plus with whole process psychological intervention provides timely psychological interventions for the patients through active communication, which helps the patients better regulate their emotions. Moreover, continuity of care plus whole process psychological intervention also resulted in significantly lower cancer-related fatigue scores and a better quality of life of patients versus routine care. Research has shown that TCM care can effectively improve the physiological condition and quality of life of lung cancer patients [18] and can be adopted in future care. The results of the present study also showed that patients given continuity of care plus whole process psychological intervention had a higher treatment compliance versus those given routine care. The reason may be that the health education and active communication in the combined nursing provide a better understanding of the disease and better psychological status of the patients, which allows for a positive feedback in terms of treatment compliance given a better life attitude of patients. This also coincides with the nursing intervention of the TCM rapid rehabilitation concept model, which can significantly shorten the postoperative recovery of lung cancer patients, improve the nutritional status, reduce the incidence of postoperative complications, and enhance the survival quality of patients [18].

It has been shown that both pharmacological and nonpharmacological approaches to alleviate depression may contribute to improving the quality of life in patients with lung cancer due to the negative consequences of the disease symptoms on quality of life. Thus, psychological screening and appropriate interventions are essential for advanced cancer care [20]. In the present study, the combined nursing also resulted in a high nursing satisfaction versus routine care, which was consistent with the existing research conclusions [20]. Continuity of care plus whole process psychological intervention can effectively mitigate the negative emotions of lung cancer patients, alleviate cancer-related fatigue, improve treatment compliance, and boost the life quality of patients.

## 5. Conclusion

Continuity of care plus whole process psychological intervention can effectively mitigate the negative emotions of lung cancer patients, alleviate cancer-related fatigue, improve treatment compliance, and boost the life quality of patients. However, as this study was a retrospective study with inclusion bias, the number of cases will be expanded in the future to conduct a multicenter, prospective, large sample size study to provide a referential basis for clinical use.

## Figures and Tables

**Figure 1:** Comparison of SES scores between the two groups.

**Figure 2:** Comparison of Morisky scores between the two groups.

**Figure 3:** Comparison of nursing satisfaction between the two groups.

**Table 1:** General data comparison between patients in two groups ($\bar{x}\pm s$).

Index	Observation group (*n* = 65)	Control group (*n* = 65)	*t*/*x*^2^	*P* value
Gender			3.265	0.415
Male	39	41		
Female	26	24		
Age (years)	(58.89 ± 12.13)	(58.76 ± 12.57)	0.06	0.952
*Pathological classification*				
Small cell lung cancer	11	9	1.236	0.366
Squamous cell carcinoma	21	19	2.365	0.145
Adenocarcinoma	27	32	1.024	0.245
Large cell carcinoma	6	5	3.415	0.365
TNM staging			4.156	0.323
III	35	32		
IV	30	33		

**Table 2:** Comparison of HAMD and HAMA scores between the two groups before and after nursing intervention ($\bar{x}\pm s$).

Groups	Number	HAMD		HAMA	
		Before nursing	After nursing	Before nursing	After nursing
Observation group	65	32.24 ± 2.87	18.25 ± 3.45	24.32 ± 3.71	12.66 ± 2.14
Control group	65	32.51 ± 2.34	25.68 ± 4.69	24.29 ± 3.65	16.73 ± 3.64
*t*-value		0.588	10.089	0.046	7.771
*P* value		0.558	＜0.01	0.963	＜0.01

**Table 3:** Comparison of cancer-related fatigue scores between the two groups ($\bar{x}\pm s$).

Groups	*n*	Physical dimension	Behavioral dimension	Cognitive dimension	Emotional dimension
Observation group	65	5.39 ± 0.13	3.08 ± 0.52	3.43 ± 0.49	4.28 ± 0.74
Control group	65	7.13 ± 1.28	4.83 ± 1.17	4.71 ± 1.23	6.23 ± 0.68
*t*-value		10.904	11.02	7.794	45.643
*P* value		＜0.01	＜0.01	＜0.01	＜0.01

**Table 4:** Evaluation and comparison of life quality in patients with lung cancer between the two groups ($\bar{x}\pm s$).

Groups	*n*	Lung cancer-specific module	Functional dimension	Social/family dimension	Emotional dimension	Physiological dimension
Observation group	65	33.70 ± 1.31	23.58 ± 3.15	25.54 ± 2.37	21.35 ± 0.49	25.32 ± 3.23
Control group	65	25.18 ± 1.62	17.24 ± 1.33	20.08 ± 1.64	17.36 ± 0.14	18.04 ± 0.39
*t*-value		32.971	14.949	15.274	63.124	18.040
*P* value		＜0.01	＜0.01	＜0.01	＜0.01	＜0.01

^∗^indicates that there are differences between the two groups.

## Data Availability

The datasets used during the present study are available from the corresponding author upon reasonable request.
